The article "Detection and Analysis of Perfusion Pressure through Measuring Oxygen Saturation and Requirement of Dural Incision Decompression after Laminectomy" was retracted in 2023. Reasons: signs of a paper mill; suspected computer-generated content; unreliable results or conclusions; lack of ethics approval or compliance.

# Detection and Analysis of Perfusion Pressure through Measuring Oxygen Saturation and Requirement of Dural Incision Decompression after Laminectomy

**DOI:** 10.1155/2021/8560668

**Published:** 2021-12-06

**Authors:** Jamal Alshorman, Yulong Wang, Guixiong Huang, Tracy Boakye Serebour, Xiaodong Guo

**Affiliations:** Department of Orthopedics, Union Hospital, Tongji Medical College, Huazhong University of Science and Technology, Wuhan 430022, China

## Abstract

**Background:**

Traumatic spinal cord injury (SCI) can continue and transform long after the time of initial injury. Preventing secondary injury after SCI is one of the most significant challenges, and early intervention to return the blood flow at the injury site can minimize the likelihood of secondary injury.

**Objective:**

The purpose of this study is to investigate whether laminectomy can achieve the spinal cord blood flow by measuring the spinal blood oxygen saturation intraoperatively without the presence of light.

**Methods:**

Between June and August 2021, eight patients were admitted after traumatic spinal cord injury for surgical treatment. We explored the effectiveness of laminectomy and whether the patients required further procedures or not. We used a brain oxygen saturation monitor at the spine injury site under dark conditions.

**Results:**

Eight cervical trauma patients, six males and two females, underwent laminectomy decompression. Three patients' ASIA grade improved by one level, and one patient showed slight motor-sensory improvement. Oxygen saturation was in the normal range.

**Conclusion:**

Performing bony decompression can show good results. Therefore, finding an examination method to confirm the improvement of blood perfusion by measuring oxygen saturation at the injury site after laminectomy is essential to avoid other complications.

## 1. Introduction

SCI is a life-threatening condition, and deciding the proper treatment method has a significant role in its prognosis. However, some patients showed substantially positive outcomes after laminectomy, while some required an additional durotomy. A primary spine injury can lead to consequential injury. This secondary injury is often catastrophic and is accompanied by a variety of complications [1]. At least 25 well-established secondary injury mechanisms can occur within minutes, weeks, and months following SCI [2]. If the probability of the occurrence of secondary injury is reduced, the loss of nerve function after SCI will be decreased and it will significantly improve the chances of regaining some lost neurological functions. Decompression surgery opens the bony canals through which the spinal cord and nerve pass, creating more space for them to move freely. The laminectomy opens a window allowing the dural sac (containing nerves) to re-expand in the space. After extensive bony decompression, cord compression against the dura may only occur in a few patients [3]. Performing durotomy with duroplasty can reduce the intraspinal pressure (ISP) and decrease the spinal cord compartment syndrome (SCCS), improving spinal cord perfusion pressure (SCPP) and blood perfusion at the injury site [4, 5]. However, to perform durotomy and duroplasty, an experienced surgeon is needed because it causes a higher risk of injury such as spinal cord swelling and cerebrospinal fluid leakage [6]. Confirming blood perfusion after performing laminectomy is essential to avoid durotomy complications and their associated risk factors. However, if decompression during laminectomy cannot release dural pressure, an additional dural incision and decompression can be done, and the cerebrospinal fluid circulation is highly likely to return.

The article "Detection and Analysis of Perfusion Pressure through Measuring Oxygen Saturation and Requirement of Dural Incision Decompression after Laminectomy" was retracted in 2023. Reasons: signs of a paper mill; suspected computer-generated content; unreliable results or conclusions; lack of ethics approval or compliance.

Spinal dural decompression can reduce intradural pressure, thereby inhibiting spinal cord swelling. The occurrence of SCCS after SCI is common and leads to poor prognosis. Dural incision and duroplasty are designed to alleviate the symptoms of this SCCS [5, 7]. With the control of SCCS and the reduction of secondary damage, patients may have better nerve recovery. When decompression is performed at the level of the dura, nerve function is significantly restored [8, 9]. The prognosis will depend on the blood flow to the damaged area. This study shows the effectiveness of measuring oxygen saturation after laminectomy and assesses whether the patients require further procedures (dural decompression). Also, this study aims to confirm the benefits and effectiveness of bony decompression on SCPP in SCI patients.

### 1.1. Laminectomy Alone versus Durotomy with Duroplasty

Durotomy helps to decompress the spinal cord thoroughly and improves CSF circulation in severe SCI; also, it decreases ISP to less than 20 mmHg. While laminectomy alone is insufficient in some cases, durotomy decompression will be needed [4, 5]. The hematoma between the dura and spinal cord can increase the pressure that cannot be relieved by laminectomy. However, durotomy with duroplasty effectively reduces ISP, improves SCPP, and microcirculation of the spinal cord; CSF pulsation will be restored [10]. Restoring normal gradients of ISP across the spinal cord enhances blood perfusion, blocking possible secondary ischemia [11]. Because of the risks associated with durotomy and its complications, examining the laminectomy procedure's effectiveness (case-by-case) before performing durotomy is essential. Finding a method to ensure SCPP improvement after laminectomy is necessary to produce a better prognosis. If the spinal cord oxygen saturation is normal after sufficient bony decompression is completed, then SCPP has improved. A dural incision decompression is not required.

The article "Detection and Analysis of Perfusion Pressure through Measuring Oxygen Saturation and Requirement of Dural Incision Decompression after Laminectomy" was retracted in 2023. Reasons: signs of a paper mill; suspected computer-generated content; unreliable results or conclusions; lack of ethics approval or compliance.

## 2. Method and Surgical Procedure

### 2.1. Inclusion and Exclusion Criteria

We have chosen the trauma patients older than 18 years old, with radiological abnormalities in the cervical region.

Between June and August 2021, eight patients underwent bony decompression and internal fixation. The operation was performed as early as possible (between 24 hours and 16 days).

After obtaining general anaesthesia, the patients were placed in the prone position, with the neck gently bent for a better view, and a head holder was used. After making a midline incision, the fascia and muscles were dissected to reveal the posterior arch. The midline incision should be more than 12 cm. We adopted the same surgical procedure: posterior laminectomy followed by oxygen saturation measurement in all patients. Before extensive laminectomy, spinal blood oxygen saturation was measured first and recorded. After extensive laminectomy, spinal blood oxygen saturation was measured and recorded again. If spinal blood oxygen saturation was not improved or remained the same as the first measurement, more extensive laminectomy or durotomy with duroplasty was needed. After an extensive laminectomy (3–4 segments), the spinal cord pulsation (CSF circulation) was observed to check the improvement of blood perfusion. The injury site was checked for the existence of hematoma by direct visualization. The probe was inserted to measure the spinal oxygen saturation about 1 cm away from the dural sac (see Figures 1 and 2). Spinal blood oxygen saturation was measured in a dark environment. After that, depending on the oxygen saturation being in normal range (58%–68%), the decision to perform durotomy or not was made. Posterior fusion was performed in all cases.

### 2.2. Working Principle

The brain oxygen monitor uses near-infrared light with a wavelength between 700 and 900 nm. Since near-infrared light has good penetrability to the skin, fat, and skull, it can penetrate the aforementioned outer tissues and detect the blood oxygen parameters of deeper brain and muscle tissues. The near-infrared light enters the tissue from the light source of the probe, passes through the tissue to be tested, and is received by the receivers at two different positions of the probe. The probe of oxygen saturation measurement will not cause any trauma or pain to the patient; there is no lag in data collection and continuous and uninterrupted data collection; there is no need to infer blood oxygen information of local tissues indirectly through the blood oxygen information of the whole body. We used this equipment to monitor spinal blood oxygen saturation directly at the injury site. This was done to investigate whether there was a change in the blood oxygen saturation of the dura mater in patients with SCI and the effect on the prognosis of the patient.

The article "Detection and Analysis of Perfusion Pressure through Measuring Oxygen Saturation and Requirement of Dural Incision Decompression after Laminectomy" was retracted in 2023. Reasons: signs of a paper mill; suspected computer-generated content; unreliable results or conclusions; lack of ethics approval or compliance.

## 3. Results

Eight patients with traumatic cervical SCI came to the Orthopedic Department of Union Hospital of Tongji Medical College for treatment. The youngest patient was 35 years old, and the oldest one was 66 (six males and two females). Physical examination and American Spinal Injury Association impairment scale were used to grade the severity of SCI. However, ASIA grades before the operation were (A in five patients, D in two patients, and C in one patient). Surgical intervention was between 24 hours and 16 days after injury. Laminectomy and vertebral body fusion were performed, and bone graft was applied.

Before extensive laminectomy, spinal blood oxygen saturation was measured first and recorded. After extensive laminectomy, spinal blood oxygen saturation was measured and recorded again. If spinal blood oxygen saturation was not improved or remained the same as the first measurement, more extensive laminectomy or durotomy with duroplasty was needed. We failed to measure oxygen saturation of one patient. Two patients were transferred to the intensive care unit after the operation and underwent a tracheotomy. On the last follow-up, the ASIA grade improved in three patients, 2 patients (A to B) and one (A to D), two remained the same (one D and one A), and one patient died; the details of other two patients are not stated here. Sensory function improved in all patients except two (the one whose grade remained the same and the one who died) (see Table 1).

## 4. Discussion

High ISP and low SCPP can cause low oxygen saturation of the spinal cord tissue, which requires surgical decompression. Finding a method to examine blood flow at the injury site is essential in every patient to predict the prognosis, ensure no other treatment method is required, and avoid other procedure complications [6]. The pressure around the spinal cord can lead to a decrease in the blood flow at the injury site that can cause ischemia of the spinal tissue [12]. Measuring the oxygen saturation at the injury site can reveal whether laminectomy is enough or not (see Figure 3).

The significance of monitoring the blood oxygen saturation of the spinal cord during the operation is as follows. (1) During the operation, the blood oxygen saturation of the spinal cord tissue at the injury site can be directly measured, which can indirectly reflect the blood perfusion pressure of the spinal cord. (2) Whether the spinal cord decompression is complete can be determined. The tissue oxygen saturation is restored or improved, indicating that the decompression is effective. (3) Guidance on whether to do more extensive lamina decompression or more thorough dural incision decompression and other operations can be given.

The article "Detection and Analysis of Perfusion Pressure through Measuring Oxygen Saturation and Requirement of Dural Incision Decompression after Laminectomy" was retracted in 2023. Reasons: signs of a paper mill; suspected computer-generated content; unreliable results or conclusions; lack of ethics approval or compliance.

Secondary injuries of SCI occur through multi-variant pathological mechanisms [2, 13]. Inflammatory process and increase in the pressure lead to tissue damage [14, 15]. Preventing secondary injury after SCI is one of the significant challenges [10, 16, 17]. However, the dura mater compressed the swollen spinal cord, leading to raised ISP and a progressive reduction of blood flow, leading to chronic hypoxia [8, 18, 19]. An appropriate treatment method is essential to decrease ISP and improve SCPP. However, performing bony decompression is not enough to reduce the pressure around the injury site. Even if bony decompression is performed early, gradually, or instantly, swelling can create subarachnoid occlusion [20]. Ensuring the blood flow circulation returns to normal is the primary purpose of predicting the prognosis in surfer SCI [21].

In brain trauma, maintenance of adequate cerebral oxygenation is critical in managing patients with brain injury; otherwise, it leads to hypoxia [22]. Maintaining the supply of oxygen and other nutrients at the injury site will end the inflammatory process from progression. Measuring the adequate oxygen delivery to a tissue depends on sufficient oxygen content in arterial blood and blood flow to the tissue utilizing pulse oximetry [23]. Also, acceptable oxygen delivery can assess susceptibility to injury and tissue damage [24].

There is a growing concern about the synergistic regeneration of bone and correlated vasculature, nerves, cartilage, tendon, ligaments, and muscles. Therefore, designing examination methods intraoperatively would open new doors to repairing and regenerating tissues after SCI [25]. Monitoring tissue oxygenation can evaluate both tissue oxygenation and microcirculation beyond macro-hemodynamic measurements [26]. Low blood flow at the injury site will cause hypoxemia (abnormally low oxygen level in tissue (<60 mmHg)) [27]. Low arterial blood oxygenation indicates a reduction in oxygen delivery due to vasospasm or hypotension or inadequate blood perfusion [28]. Measuring the spinal blood oxygen saturation can provide information about blood perfusion [29]. Measuring the spinal oxygen saturation in dark conditions is done because the light can affect the examination results. However, this method is based on light transmission in the near-infrared spectrum across tissue and its absorption [30]. Measuring spinal blood oxygen saturation can help the clinician justify the change in the treatment method to influence potential deficiencies and the requirement of other procedures in every patient [6, 31].

The article "Detection and Analysis of Perfusion Pressure through Measuring Oxygen Saturation and Requirement of Dural Incision Decompression after Laminectomy" was retracted in 2023. Reasons: signs of a paper mill; suspected computer-generated content; unreliable results or conclusions; lack of ethics approval or compliance.

Before decompression, we found that the oxygen saturation of spinal cord tissue was low, which may be caused by high ISP and low SCPP. We emphasized the need for surgical decompression and other interventions. There are many ways to determine decompression during operation, the level of decompression, cerebrospinal fluid pulsation, or blood circulation recovery. However, laminectomy decompression is empirical and cannot accurately determine the CSF circulation recovery. Simultaneously, these methods cannot directly reflect the situation of spinal cord tissue oxygen saturation. The significance of intraoperative monitoring of spinal cord oxygen saturation is as follows: direct measurement of the spinal cord blood oxygen saturation can indirectly reflect the blood perfusion pressure; whether the decompression is complete or not and the oxygen saturation of spinal cord tissue is restored or improved can be determined, indicating that decompression is effective; and guidance on whether to do a wider range of lamina decompression or more thorough dural incision decompression and other operations can be given.

Moreover, performing further procedure in case of abnormal oxygen saturation can affect the specific physiological deficit and hasten the healing of the injury. This can also make medical care decisions more personal and tailored to each case, minimizing unnecessary interventions and making patient follow-up easier. Also, this strategy can increase the chances of improving the current medical practice. Further monitoring tissue oxygenation can evaluate blood perfusion and confirm whether laminectomy is enough or the patient will need further durotomy. If the oxygen saturation is in the normal range, laminectomy will be enough to achieve significant outcomes, while if it is abnormal, then bony decompression is not enough to reduce ISP and improve the SCPP, requiring durotomy.

Oxygen saturation measurement equipment can be used for

1. Monitoring the oxygen metabolism of the patient's spine tissue.
2. Assisting the clinical realization of noninvasive and continuous monitoring of spinal oxygen saturation.
3. Early detection of hypoxia and ischemia in the patient's spine tissue.
4. Judging short-term neurodevelopmental prognosis.
5. Evaluation of the safety and effectiveness of the clinical treatment plan.
6. Assisting in evaluating the degree of SCI.

The article "Detection and Analysis of Perfusion Pressure through Measuring Oxygen Saturation and Requirement of Dural Incision Decompression after Laminectomy" was retracted in 2023. Reasons: signs of a paper mill; suspected computer-generated content; unreliable results or conclusions; lack of ethics approval or compliance.

In these cases, the oxygen saturation was normal. We did not perform dural decompression as the SCPP improved at the injury site. Many factors affect the prognosis of the SCI, including severity of the injury, time of surgery, hematoma, and edema. Measuring spinal blood oxygen saturation is essential to confirm the improvement of SCPP after laminectomy. We failed to measure the oxygen saturation in one patient because the patient was thin and short, and we could not make the incision longer than 12 cm, so the space for the probe was not enough.

## 5. Limitations

This study has some limitations. First, this study evaluated a limited and small number of cases. Eight patients were involved and underwent spinal blood oxygen saturation measurement, and one of them failed the oxygen measurement. Second, spinal blood oxygen saturation was within normal range in all patients after laminectomy. Third, we chose only the patients with cervical abnormalities. In addition, the follow-up time is short for confirming the improvement after laminectomy. This is to say, more oxygen saturation measurement cases are thus needed.

## 6. Conclusion

Treating SCI patients with bony decompression can achieve significant outcomes but not in all cases. Decreasing the pressure around the injured spinal cord and increasing the blood flow are the mainstay interventions to achieving better results. Detecting the improvement of SCPP at the injury site is essential to confirm the benefit of laminectomy. Spinal blood oxygen saturation measurement under dark conditions might help in deciding whether to perform further procedures (durotomy with duroplasty or extensive laminectomy) or not. By monitoring spinal cord oxygen saturation in real time throughout the operation, it is possible to monitor the spinal cord perfusion pressure.

## Figures and Tables

**Figure 1:** (a, b) Laminectomy procedure and spinal blood oxygen saturation measurement under dark conditions during the operation. (c) The probe. (d) The intraoperative display indicating that the spinal blood oxygen saturation is 68.3%.

**Figure 2:** 66-year-old male with ASIA grade D underwent laminectomy and spinal blood oxygen saturation measurement. (a) Preoperative MRI. (b) C3–C6 bony decompression. (c) Insertion of the probe for oxygen saturation measurement. Oxygen saturation measurement failed in this patient.

**Figure 3:** (a) An old male admitted to hospital for “head injured by a heavy object” (ASIA grade A) (diagnosis: spinal cord injury and cervical spine fracture). (b) Oxygen saturation probe was inserted after C2–C6 lamina decompression and internal fixation. (c) Spinal blood oxygen saturation was in a normal range (68.3%). Postoperative ASIA grade improved to grade D.

The article "Detection and Analysis of Perfusion Pressure through Measuring Oxygen Saturation and Requirement of Dural Incision Decompression after Laminectomy" was retracted in 2023. Reasons: signs of a paper mill; suspected computer-generated content; unreliable results or conclusions; lack of ethics approval or compliance.

**Table 1:** A clinical summary of patients (laminectomy followed by spinal blood oxygen saturation measurement).

Cases	Age	Gender	Injury mechanism	Operation level	ASIA (preoperative)	ASIA (postoperative)	Time of operation	Oxygen saturation
1	35 y	M	Fall	C2–C6	D	D	102 hours	Normal
2	55 y	M	Fall	C2–C6	A	B	24 hours	Normal
3	64 y	F	Fall	C3–C5	A	A	30 hours	Normal
4	58 y	M	Fall	C3–C6	A	Died	24 hours	Normal
5	52 y	F	Fall	C3–C6	A	B	64 hours	Normal
6	57 y	M	Head injury by heavy object	C2–C6	A	D	29 hours	Normal
7	56 y	M	RTA	C3–C6	C	—	3.18 hours	Normal
8	66 Y	M	NS	C3–C6	D	—	16 days	Failed to measure

ASIA impairment scale: American Spinal Injury Association impairment scale; M: male; F; female; RTA: road traffic accident.

## Data Availability

The patients' history and other data used to support the findings of this study are available from the corresponding author upon request.
